This article has been retracted.

# Evaluation of Urban Tourism Carrying Capacity Based on Analytic Hierarchy Process Optimizing BP Neural Network

**DOI:** 10.1155/2022/5991381

**Published:** 2022-05-16

**Authors:** Jia Li, Yuan Wang

**Affiliations:** ^1^College of History, Culture and Tourism, Sichuan Normal University, Chengdu 610066, Sichuan, China; ^2^College of International Education, Sichuan Normal University, Chengdu 610066, Sichuan, China

## Abstract

With the rapid development of today's social economy, tourism has also developed rapidly. According to national statistics, from 2017 to 2019, domestic tourism revenue increased from 4.57 trillion to 5.73 trillion. The tourism economy has made more and more contributions to the national economy, and it has also received more and more attention and attention from society. However, in recent years, the “explosive” growth of tourism has not only promoted economic development but also brought some challenges to society and the economy, such as environmental pollution in tourist cities. Therefore, it is of great significance to evaluate the tourism carrying capacity of a tourist destination city to realize the sustainable development of the city's tourism. This article aims to study the evaluation of urban tourism carrying capacity based on AHP and an optimized BP neural network. It designs a carrying capacity evaluation system, conducts BP neural network training for the system, and conducts system testing. The results show that the proportion of scientific and technological innovation is obviously higher than that of other aspects in the proportion of carrying capacity indicators in various aspects of each city. Environmental carrying capacity indicators can be divided into resource supply indicators, pollutant containment indicators, and social impact indicators. This article divides the important indicators into economic development, technological innovation, potential competition, environmental support, and development guarantee. Its indicators account for about 50%, with an average of more than 40%. This shows that the system can clearly display the main factors and evaluation indicators that affect the urban tourism carrying capacity and has certain feasibility and reliability.

## 1. Introduction

With the development of the global social economy and the improvement of people's living standards, people are more and more keen on tourism, which has made the tourism industry continue to develop rapidly. From 2017 to 2019, the number of domestic tourists increased from 5.001 billion to 6.006 billion, according to national statistics. The rapid development of tourism plays a self-evidently important role in promoting economic development and promoting the urbanization development process of destination cities. Therefore, tourism has received more and more attention from the state and society. In recent years, the explosive growth of domestic and foreign tourism has brought many problems and challenges while promoting the economic development of various countries and regions. For example, in terms of economy, the economic development of a country or city is overly dependent on tourism. Socially, the increasing influx of tourists into tourist destination cities has resulted in increased pressure on the city's population and traffic management. It will also easily lead to the escalation of conflicts between tourists and local residents and will also cause certain pollution to the local environment. In terms of culture, the input of tourists' culture is likely to have a certain impact on the local traditional culture of the destination city and so on. These issues and challenges can have a huge negative impact on the sustainable development of the local tourism industry and may cause the city's tourism industry to reach or exceed growth limits or even decline. Therefore, these overtourism phenomena that exceed the tourism carrying capacity of tourist destination cities should be highly valued by the country and society. In order to ensure and promote the sustainable development of tourism, it is necessary and urgent to evaluate a city's tourism carrying capacity. Analytic hierarchy process is a decision-making method that decomposes decision-related elements into specific programs and conducts qualitative and quantitative analysis on this basis. The optimized BP neural network is an improved multilayer feedforward neural network trained according to the error backpropagation algorithm, and it is also one of the most widely used neural network models. The combination of AHP and an optimized BP neural network can play a certain role in the evaluation of a city's tourism carrying capacity. Therefore, this article mainly studies how to evaluate urban tourism carrying capacity based on AHP and optimized BP neural network. The optimized BP neural network can process and analyze data more quickly, and the analytic hierarchy process can more intuitively reflect the important indicators of urban tourism environment carrying capacity.

The innovations of this article are as follows: (1) it has carried out research on the evaluation of urban tourism carrying capacity that is lacking in the academic world; (2) it combines the AHP and the optimized BP neural network algorithm to carry out the experimental research on the urban tourism carrying capacity and draws effective conclusions.

## 2. Related Work

Since AHP and optimized BP neural network have high application value in many fields, such as biomedicine, Internet of Things, and computer science, many researches related to AHP and optimized BP neural network have emerged in the academic circles. Among them, Abdelazim A I's research focused on the application of AHP in building energy efficiency rating system. He proposed a new building energy efficiency rating system based on the AHP standard [1]. Jagtap H P mainly studied the application of AHP in the identification of key equipment in thermal power plants. In his research, he considered the impact of key equipment failures in thermal power plants on power generation, environment and safety, failure frequency, and maintenance costs based on AHP [2]. Singh et al. studied the optimization effect of AHP on the design problem of automatic generation controller for multiregional power systems. They carried out the controller design and performance analysis based on AHP [3]. Arif W. M. mainly studied the training and optimization of deep learning neural network models based on the optimized BP neural network. He proposed a new method for supervised fine-tuning of deep network models [4]. Zhao et al. studied the application of an optimized BP neural network in the prediction of flexural strength of open-cell composites. It is proved by experiments that the prediction model proposed by them based on the optimized BP neural network has good prediction accuracy [5]. He F. mainly studied the application of an optimized BP neural network in the prediction of phosphorus content in molten steel at the end of steelmaking. He also combined the method of clustering and predicting a two-stage mixture to carry out experimental prediction analysis [6]. Although the above researches are closely related to the tomographic analysis method and the optimized BP neural network, the experimental process of these researches is relatively complicated and difficult to operate.

## 3. Evaluation Method of Urban Tourism Carrying Capacity

### 3.1. AHP

Analytic hierarchy process (AHP) is a method of problem analysis using hierarchical logic. It can stratify and quantify people's thinking process and use mathematical analysis, decision-making, or control to provide a quantitative basis. It is suitable for decision analysis processes that are both quantitative or qualitative. It is an effective method for systematic analysis and scientific decision-making. AHP means that when analyzing a problem, the layers are firstly specified and layered, and then a hierarchical organization model is established. AHP decomposes the problem into different components according to the nature of the problem and the overall goal to be achieved and aggregates and combines the factors at different levels according to the interrelated influence and affiliation between the factors to form a multilevel analysis structure model, so that the problem ultimately boils down to the determination of the relative importance of the lowest level (plans, measures, etc. for decision-making) relative to the highest level (total goal) or the relative order of relative importance. It goes through a hierarchical model so that the research question will consist of several elements. These elements form a hierarchy according to the logical relationship, which can generally be divided into three categories: the highest layer, the middle layer, and the lowest layer. The AHP is specifically divided into four steps, namely, the creation of a ladder hierarchy model, the creation of each judgment matrix in each layer, the single-level sorting, and the total sorting and consistency check [7, 8]. AHP takes the research object as a system and makes decisions according to the way of thinking of decomposition, comparison and judgment, and synthesis. It has become an important tool for system analysis developed after mechanism analysis and statistical analysis. The idea of the system is not to cut off the influence of each factor on the result, and the weight setting of each layer in the AHP will ultimately affect the result directly or indirectly, and the degree of influence of each factor in each layer on the result is the same, quantitative, very clear, and unambiguous. This method is especially useful for systematic evaluations of unstructured properties and multiobjective, multicriteria, multiperiod systematic evaluations. The model framework of AHP is shown in Figure 1.

The basic steps of AHP are as follows.

It first determines the problem and related factors, analyzes the related factors of the problem, and judges the priority of the factors. After collecting all relevant data, it uses the AHP to carry out a logical hierarchical analysis of the structure of the problem. It assigns relevant factors to different target layers, criterion layers, and scheme layers. After the hierarchical model is established, the scale and pairwise comparison judgment matrix can be constructed. It first calculates the weight of a single element through the pairwise judgment matrix of B. To get its weight vector, it can be solved by the method of solving the characteristic root [9, 10]. It establishes the following characteristic formula:

(1) $$\begin{array}{c} B\mu =\gamma_{\max}. \end{array}$$

Among them, B is a judgment matrix, which is the eigenvector corresponding to the largest eigenroot in the matrix, and represents the largest eigenvalue in the matrix. For the judgment matrix B, if the matrix is consistent, standardize the factors of each row to obtain the exact value of the weight vector. If the matrices are inconsistent, normalizing the factors in each row yields a vector approximation of the weights. The weighted average calculation is performed on the standardized weight vector to obtain the final value of the weight vector, which is as follows:

(2) $$\begin{array}{c} \mu_{i}=\frac{\sum_{i=1}^{n}b}{\sum_{k=1}^{n}b_{ki}}. \end{array}$$

Among them, *μ*_*i*_ is the weight of the ith factor, and *n* is the order of the judgment matrix B. The eigenroot corresponding to the eigenvector is calculated as follows:

(3) $$\begin{array}{c} \gamma_{\max}=\sum_{i=1}^{n}\frac{B\mu }{n\mu_{i}}, \end{array}$$

where *μ* is the weight vector. The next step is to calculate the root method. The same is to normalize the vectors in each row of matrix B. The difference is that the geometric mean operation is first performed on each row vector to obtain the sum of the products and then normalized as above to obtain the weight vector, which is as follows:

(4) $$\begin{array}{c} \mu_{i}=\frac{\prod_{i=1}^{n}b}{\sum_{i=1}^{n}\gamma }. \end{array}$$

However, due to the large one-sidedness and limitation of people's cognition, in practical application, it is still necessary to test whether the distribution of weights is reasonable or not. That is, a consistency test is still required, and the following three indicators are used for evaluation:

The first is the consistency indicator:

(5) $$\begin{array}{c} \text{CI}=\frac{\gamma_{\max}-n}{n-1}, \end{array}$$

where *n* is the order of the judgment matrix. The second is the consistent average stochastic RI. The consistency average stochastic index RI changes according to the change of the judgment matrix order. This value is obtained by repeatedly calculating the corresponding eigenvalues and then calculating the arithmetic mean.

And finally, the relative consistency indicator is as follows:

(6) $$\begin{array}{c} \text{CR}=\frac{\text{CI}}{\text{RI}}\gamma . \end{array}$$

When CR < 0.1, the consistency of the matrix is considered to meet the requirements, and the calculated weight vector can be accepted. Conversely, if CR > 0.1, it is considered that the matrix consistency does not meet the requirements. It needs to analyze the values in the matrix, regive the scale values of each factor, and then check and calculate until the consistency requirements are met.

The above is the basic process of the whole AHP. The basic process of AHP can be shown in Figure 2.

AHP is widely used in scientific management and decision-making in economics, science and technology, culture, military, and environment. It is often used to solve problems such as comprehensive evaluation, program decision-making, and input allocation. The tomographic analysis method was initially used in safety and environmental science, such as highway traffic safety evaluation and aviation safety evaluation in the field of traffic safety evaluation. Hazardous chemicals evaluations were conducted in the field of safety production science and the use of AHP in the field of environmental science to screen air pollution prevention and control measures and establish a multilevel water environment safety evaluation system [11, 12].

### 3.2. BP Neural Network

BP neural network is a multilevel feedforward neural network formed according to error backpropagation. It consists of an input layer, an output layer, and one or more hidden layers. Feedforward neural network is simple in structure and widely used and can approximate any continuous function and square-integrable function with arbitrary precision. And it can accurately implement any finite set of training samples. From a system point of view, a feedforward network is a static nonlinear mapping. Complex nonlinear processing capabilities can be obtained through composite mapping of simple nonlinear processing units. Each level is composed of multiple neurons that can be computed in parallel. Neurons in the same layer are not connected in any way, and the neuron nodes between layers are fully interconnected. BP neural network is the simplest and most representative neural network. BP neural network has the advantages of simple calculation and fast learning speed [13, 14]. BP neural network is a multilayer feedforward neural network trained according to the error backpropagation algorithm, and it is one of the most widely used neural network models. Its outstanding advantages are its strong nonlinear mapping ability and flexible network structure. The number of intermediate layers of the network and the number of neurons in each layer can be arbitrarily set according to the specific situation, and the performance varies with the difference in the structure.

The basic principle of the BP neural network algorithm is as follows: first, the input vector is passed from the neurons in the input layer to the neurons in the hidden layer. In the hidden layer, the information is processed and transformed through the combined action of weights, thresholds, and activation functions and then passed to the output layer. An activation function is a function that operates on the neurons of an artificial neural network and is responsible for mapping the input of the neuron to the output. The activation function is introduced to increase the nonlinearity of the neural network model. Each layer without an activation function is equivalent to matrix multiplication. Even if you stack several layers, it is nothing more than a matrix multiplication. The output layer is responsible for processing the data out and making adjustments. In the process of forward and backward propagation, repeated network learning and training are carried out to gradually adjust and improve the network performance. When the set error accuracy or the maximum number of iterations is reached, the training is terminated, which means that the network has converged [15, 16]. Convergence is an economic and mathematical term and an important tool for studying functions. It refers to converging at a point and approaching a certain value. Convergence types include convergent sequence, function convergence, global convergence, and local convergence.

The basic implementation steps of the BP neural network algorithm are as follows:

(1) It initializes the weights and thresholds of the network. That is, all network connection weights *w* and threshold *b* are set to a random number within the range of [−1, +1];
(2) It is given a set of network training samples, which contains the input vector P and the expected output result *R*;
(3) It calculates the output values of the hidden layer and the output layer according to the formula; The output value of the hidden layer is as follows:
  (7) $$\begin{array}{c} a_{1}=f1\left(\sum_{i=1}^{r}\mu p_{i}+b_{1}\right). \end{array}$$
  (i) The output of the output layer is as follows:
    (8) $$\begin{array}{c} a_{2}=f2\left(\sum_{i=1}^{s1}\mu 2+b_{2}\right), \end{array}$$
  (ii) where *f*1 and *f*2 represent the activation functions defined by the input layer to the hidden layer and from the hidden layer to the output layer, respectively.
(4) Reverse error correction weight is as follows:

The error between the actual output of the network and the expected output is as follows:

(9) $$\begin{array}{c} E=\frac{1}{2}{\left(D-F\right)}^{2}, \end{array}$$

which is

(10) $$\begin{array}{c} E=\frac{1}{2}\sum_{k=1}^{I}{\left(D_{k}-F_{k}\right)}^{2}. \end{array}$$

The functional relationship between error and weight is as follows:

(11) $$\begin{array}{c} E=\frac{1}{2}\sum_{k=1}^{I}\left(d_{k}-f_{2}\sum_{j=0}^{i}f_{1}\sum_{i=0}^{n}\right). \end{array}$$

It can be seen from the above formula that the size of the error can be changed by adjusting the weights. The adjustment amount of each neuron's weight is equal to the learning rate multiplied by the negative gradient of the error function [17, 18]. The weight adjustment process from the hidden layer to the output layer is as follows:

(12) $$\begin{array}{c} \Delta W_{\text{jk}}=-\frac{\partial E}{\partial W_{\text{jk}}}, \end{array}$$

which is as follows:

(13) $$\begin{array}{c} \Delta W_{\text{jk}}=-\frac{\partial E}{\partial \;{\text{net}}_{k}}y_{j}. \end{array}$$

It sets the error signal from the hidden layer to the output layer to *ρ*_*k*_, then

(14) $$\begin{array}{c} \rho_{k}=-\frac{\partial E}{\partial \;{\text{net}}_{j}}, \end{array}$$

which is

(15) $$\begin{array}{c} \rho_{k}=d_{k}-f_{2}\left({\text{net}}_{k}\right). \end{array}$$

In this way, the weight adjustment amount from the hidden layer to the output layer can be obtained as follows:

(16) $$\begin{array}{c} \Delta V_{\text{jk}}=\left(d_{k}-f_{k}\right)f_{2}y_{j}. \end{array}$$

The parameter adjustment process of the entire BP neural network algorithm is shown in Figure 3.

## 4. Evaluation System of Urban Tourism Carrying Capacity

### 4.1. Design of Evaluation System

Urban tourism resources are composed of various types of tourist attractions (spots). And they vary in size, quality, and location. It can be seen that the carrying capacity of the tourism environment has nonequilibrium and spatial differences. Spatial differences refer to the differences in the level of social and economic development and its structure in different regions, and balance refers to the matching of environmental carrying capacity and tourism conditions.

The evaluation of tourism environment carrying capacity is through specific indicators. It predicts and guides the development trend of tourism activities in a certain period and specific tourist destinations. It continuously improves the quality of the environment while enhancing the effectiveness of tourism management activities. The early system of the carrying capacity of the tourism environment is a complex system composed of many factors such as nature, economy, and society. This is based on the theory of sustainable development, through certain technical methods, to analyze the indicators reflecting the carrying capacity of the tourism environment. It evaluates the tourism environment and the operation of the tourism environment system to prevent deviation from the normal track and achieve the coordinated development of the tourism economy and social environment [19].

In order to scientifically and rationally regulate the urban tourism environment system and timely reflect the utilization of resources and environment by tourism so as to keep it at a reasonable scale of tourism development, this article introduces the concept of urban tourism environment carrying capacity. It refers to the alarm established by the tourism industry for the development and utilization of urban natural ecotourism resources and social and cultural tourism resources under overloaded or underloaded situations. The weak urban tourism environment indicates that tourism resources have not been fully and effectively utilized, resulting in idle and waste of tourism resources. The overload of the urban tourism environment reflects that the development and utilization of tourism resources in urban tourism exceed the range that the environment can bear.

The functions of the urban tourism environment carrying capacity system include evaluation and monitoring. It is an effective way to diagnose and monitor the development status and future evolution trends of the urban tourism environment. The existence of the system aims to achieve relative stability and balance among the various influencing factors of the urban tourism environment carrying capacity. This enables it to meet the tourist's sightseeing and entertainment needs without irreversibly negatively affecting and damaging the environment. It predicts tourism environmental risks and excludes factors that damage the tourism environment. It ensures that the urban tourism environment system is in a relatively stable and benign operation and ultimately realizes the healthy and sustainable development of the urban tourism environment and local tourism [20].

The urban tourism environment carrying capacity evaluation system takes the urban tourism environment carrying capacity in the process of tourism development as the research object. The system releases information on the current situation of the tourism environment in a timely and regular manner, diagnoses whether the tourism environment deviates from the normal operating track, and thus discovers potential environmental risks as early as possible. It can also put forward corresponding control measures in response to the police situation and timely correct the original unreasonable or wrong policies and policies. It has formulated scientific, reasonable, and practical tourism environment development policies and measures. This will solve the problem of the tourism environment and realize the healthy and sustainable development of urban tourism [21].

Figure 4 is the design diagram of the urban tourism environment carrying the capacity evaluation system model designed in this article. The system mainly includes an evaluation model, data input and output, and tourism sustainable development plan.

### 4.2. Experimental Test of the Evaluation System

#### 4.2.1. Selection of Sample Data

This article selects 12 “countries and pilot cities” determined by the National Tourism Administration as online learning samples, including different regions and scenic spots in different provinces and cities. Due to the geographical proximity, the homogeneity of scenic spots, and the similarity of development levels, the samples selected in this article represent the quantitative evaluation and analysis objects. This allows for better training samples and makes the evaluation results more convincing. The way to obtain each index is shown in Table 1. The indicators are divided into A, B, and C types.

Among them, the specific sources of the index sample data of types A, B, and C are shown in Table 2.

The resource attraction and monopoly of scenic spots of different levels are shown in Table 3.

The evaluation grades of urban tourism competitiveness and the corresponding assignment rules are shown in Table 4.

#### 4.2.2. BP Neural Network Training Process

In this article, the MATLAB data processing tool is used for data training, and a total of four groups of training are carried out. In total, 5000 datasets are trained each time, and the training fitting results are shown in Figures 5 and 6. The abscissa represents the training dataset, and the ordinate represents the training data value.

#### 4.2.3. Training Results

After training with the above data, it can be seen from the figure that the fitting errors of the first and second groups of training are still relatively large. The training fitting effect of the third group is already very good, which can basically meet the calculation requirements. After the fourth group of training, the error is basically small. The two data lines almost overlap, which can be said to fully meet the calculation requirements. In order to more accurately reflect the training error of the neural network, this article makes statistics on the size of the error, as shown in Figures 7 and 8.

It can be seen from Figures 7 and 8 that the error comparison of these four groups of training. The squared value of the first group of errors is up to more than 200, and the squared value of the second group of errors is less than 100. The third group has a maximum of 30, and the fourth group of error squares has a maximum of only 10. Its training accuracy is very high, which fully meets the computational requirements.

Accordingly, the trained BP neural network is used to evaluate the urban tourism carrying capacity. The evaluation indicators mainly focus on the city's economic development, technological innovation, potential competition, environmental support, and development guarantees. It selects the key tourist attractions of the four major domestic cities of C1, C2, C3, and C4 for data statistics and analysis and evaluates their carrying capacity.

### 4.3. Experimental Results

According to the above experimental methods, the index values of all aspects of the four major cities are finally obtained, as shown in Figure 9.

It can be seen from Figure 9 that among the city's carrying capacity indicators, technological innovation accounts for the largest proportion. Among them, the scientific and technological innovation index value of C1 cities reached 0.47, which is much higher than other indicators. The second is economic development, while the environmental support is relatively weak. Therefore, in future tourism construction, it is necessary to give full play to the advantages of scientific and technological innovation and at the same time learn from each other's strengths to make up for the shortcomings in order to have more tourism carrying capacity.

Figure 10 shows the proportion of indicators in each city. It can be clearly seen from the figure that the proportion of technological innovation in the four cities is obviously higher than that of other aspects. Its indicators account for about 50%, with an average of more than 40%.

## 5. Discussion

Human activities have put too much pressure on the tourism environmental system in recent years. For example, the continuous planning and development of new tourist attractions, the dynamic changes of the environmental system itself, or the increase in the tourism area of water bodies due to natural reasons will all cause changes in the carrying capacity of the tourism environment. Its changes include both quality and quantity. The qualitative change is manifested in the change of the index system of tourism environment carrying capacity. The change in quantity is manifested as a change in the size of the indicator value.

From a theoretical point of view, the research results mainly make breakthroughs in the construction and research of the index system of urban tourism environment carrying capacity and carry out relevant case analysis. This can not only promote the further improvement of the tourism environment and tourism sustainable development theory but also have important reference significance for the research of tourism in various cities [22].

From a practical point of view, the research results can provide a safe and systematic channel and approach for the transmission of tourism environmental information. It provides precise and specific data information and technical support for urban tourism environment research. This provides a systematic and comprehensive guarantee for the city's tourism environment capacity management and also provides scientific guidance for the practice of urban tourism sustainable development strategy.

The research on cities in this article is mostly focused on the carrying capacity of sustainable development. Research on the optimization of the BP neural network urban tourism environment carrying capacity evaluation system based on AHP is relatively rare. Although some contents are involved, most of them focus on the research of concept connotation, evaluation system, quantitative model, and so on. It does not carry out special, comprehensive, and in-depth research and discussion on the urban tourism environment carrying capacity system.

## 6. Conclusion

This article firstly summarizes the research purpose and content in the abstract section. It introduces the background meaning of this article and some key contents in the introduction section. Secondly, in the related work part, this article lists some research results of some scholars related to the main content of this article so as to understand the current situation of urban tourism and the areas to be improved.

In the theoretical research part, this article firstly introduces the AHP, including its concept, model framework, and basic steps. Secondly, it introduces BP neural network, including its concept, basic principle, and process. Finally, it introduces the evaluation system of urban tourism.

In the experimental test, this article selects multiple “countries and pilot cities” determined by the National Tourism Administration as the neural network learning samples. After multiple groups of training, a neural network model with high accuracy is obtained, and the model is used to evaluate the carrying capacity of multiple cities in many aspects. The results show that the urban tourism carrying capacity evaluation system optimized by BP neural network based on AHP can more intuitively reflect the main factors included in the carrying capacity evaluation.

## Figures and Tables

**Figure 1:** AHP model architecture.

**Figure 2:** Basic flowchart of secondary analysis method.

**Figure 3:** BP neural network algorithm parameter adjustment flowchart.

**Figure 4:** Design diagram of urban tourism environmental carrying capacity evaluation system.

**Figure 5:** Fitting graph of the first two training data. (a) The first set of training; (b) the second set of training.

**Figure 6:** Fitting diagram of the third and fourth groups of training data. (a)The third set of training; (b)the fourth group of training.

**Figure 7:** The first and second sets of training squared differences.

**Figure 8:** The third and fourth groups of training squared differences.

**Figure 9:** Comparison of carrying capacity index values of various cities.

**Figure 10:** Proportion of carrying capacity indicators in various aspects of the city.

**Table 1:** How to obtain indicator data.

Index	Variable	Data sources	Kind
Foreign exchange income from tourism (billion US dollars)	*X*1	Annual statistical yearbook of tourism in various cities	A
Total tourism revenue (100 million yuan)	*X*2	Annual statistical yearbook of tourism in various cities	A
Total number of domestic and foreign tourists (10,000 person-times)	*X*3	Annual statistical yearbook of tourism in various cities	A
Construction of tourism public service platform	*X*4	Grading according to relevant standard grades	B
Development security	*X*5	The official website of the National Tourism Administration, the official tourism website of each city, and the statistical bureau of each city	B
Environmental support	*X*6	The official website of the National Tourism Administration, the official tourism website of each city, and the statistical bureau of each city	B
Potential competitiveness	*X*7	The official website of the National Tourism Administration, the official tourism website of each city, and the statistical bureau of each city	B
Technological innovation	*X*8	The official website of the National Tourism Administration, the official tourism website of each city, and the statistical bureau of each city	B
Economic development	*X*9	The official website of the National Tourism Administration, the official tourism website of each city, and the statistical bureau of each city	B
Other	*X*10	Web search	C

**Table 2:** Specific sources of sample data for different types of indicators.

Kind	Specific source
A	Statistical bulletin of national economic and social development of cities, urban statistical yearbook
B	The official website of each city's tourism, the official website of the National Tourism Administration
C	Experts in various fields assign scores to qualitative indicators according to relevant standards, web search

**Table 3:** Scenic spot resource attraction and monopoly scoring rules.

Evaluation indicators	Evaluation basis	Score
Natural resource attractiveness	World natural and cultural heritage	10
	National historical and cultural city	9
	5A-level scenic spot	8
	National key scenic spot	7
	Excellent tourist city in China	6
	National nature reserve	5
	National park	4
	Other	0

Monopoly degree of tourism resources	Rare in the world	10
	Country rare	5
	Provincial rare	2
	Other	0

**Table 4:** Evaluation level of urban tourism competitiveness and its assignment rules.

Evaluation level	Core competitiveness	Output result value
SS	Advantage	80–100
S	Strong	60–80
TT	Relatively strong	50–60
T	Medium	40–50
UU	Generally	20–40
U	Weak	1–20

## Data Availability

No data were used to support this study.
